# AHP-FSE-Based Risk Assessment and Mitigation for Slurry Balancing Shield Tunnel Construction

**DOI:** 10.1155/2022/1666950

**Published:** 2022-06-13

**Authors:** Kang Li, Xiaer Xiahou, Hong Huang, Lingyi Tang, Jie Huang, Qiming Li, Ping Feng

**Affiliations:** ^1^Department of Construction Management and Real Estate, School of Civil Engineering, Southeast University, Nanjing 211189, China; ^2^China Construction Eighth Engineering Division Corporation, Ltd, Shanghai 200112, China

## Abstract

Slurry balancing shield construction is a method in which slurry pressure and groundwater pressure are balanced to achieve stability of excavation working face. It is widely used in tunnel construction due to its safety and high-efficiency characteristics. At present, research on safety risk management of slurry balancing shield construction is relatively lacking, and most scholars still mainly focus on technical research. In this paper, based on system engineering theory and from the perspective of whole construction process, a comprehensive evaluation index system for shield construction risk analysis is built by taking “human-machine-material-method-environment” as assessment dimensions. This paper modifies the existing analytic hierarchy process (AHP), combines AHP with fuzzy synthetic evaluation to build a risk analysis model, and quantifies the construction risk by evaluation set and matrix. Combined with case study, the effectiveness of the proposed model is verified, and measures to mitigate safety risks of slurry shield construction are proposed from perspectives of management, economy, and technology. This paper evaluates the overall risk level of project from a systematic perspective, which is an extension of traditional technology-oriented research.

## 1. Introduction

Acceleration of urbanization increasingly reduces available ground space, and the development of underground space has become an important ways to expand living space. From the perspective of construction methods, cofferdam excavation and mining method has been unable to meet the current needs of underground space construction, and sinking pipe and shield tunneling method have gradually become popular. With the improvement of mechanical manufacturing level, the diameter of shield tunnel is gradually increasing, and the length of single tunneling, buried depth, and complex geological conditions are constantly setting new records. At the same time, with the extensive use of shield method, safety accidents also emerge in endlessly, work surface collapse, gushing sands and water; workers trapped problems occurred frequently; and reasons can be attributed to lack of operation and management experiences, poor mechanical equipment reliability, complex hydrogeological conditions, and so on [1–4]. Safety management and risk control of shield tunneling have become a new research topic.

Slurry balancing shield is an excavation method, which balances the pressure generated by slurry silo with the pressure of water and soil in working face, so as to maintain the stability of excavation face [5]. Research on risk control of slurry shield construction is still in its infancy. Most of existing researches are oriented to key technologies, such as ground settlement control [6–9], numerical simulation of tunnel excavation process [10, 11], influence of shield tunneling that go through existing structures [12–16], and with less research on safety risk control [17–20]. In fact, it is of great significance to improve the safety of slurry shield construction to clarify the composition of safety risks and carry out safety management from the beginning of whole life cycle of project. Analytic hierarchy process (AHP) is a common method in risk analysis research, which has irreplaceable advantages in constructing risk analysis index system and clarifying the weight of risk factors, and has been widely used in the field of civil engineering construction risk analysis [21–24]. AHP method also has strong subjectivity for qualitative and overreliance on expert opinions. Therefore, this paper introduces fuzzy synthetic evaluation to improve traditional AHP, constructs comment set and judgment matrix, and realizes the risk quantification based on the result of factor weight analysis, trying to provide mathematical basis for safety management of slurry shield construction from qualitative to quantitative, so as to precontrol safety risks in the early stage of project.

In view of current lack and deficiency of shield construction safety risk research, according to its construction process, this article demonstrates formation mechanism of construction safety risk, using analytic hierarchy process (AHP) combined with fuzzy synthetic evaluation method to carry out risk identification and evaluation. Risk factors are screened and restructured; then, evaluation model is established on this basis, and value of each risk factor is determined by risk matrixes. At the same time, taking Nanjing Metro Line 3 cross-river tunnel project as a research case, the effectiveness of proposed risk assessment method is verified, and countermeasures face to various safety risks and hidden dangers are mainly expounded from aspects of management, economic, and technology.

The remaining parts of the paper are organized as follows. Section 2 summarizes the current research on slurry shield construction technology and risk management. Section 3 constructs a construction safety risk evaluation model based on AHP-FSE method. Section 4 is a case study and quantifies construction safety risk value of a cross-river tunnel. Section 5 puts forward risk mitigation measures from multi-aspects. Section 6 makes a conclusion and discusses the future research direction.

## 2. Literature Review

Shield tunneling, as a popular method used in large-scale underground construction, is playing an increasingly important role in urban metro, cross-river tunnel, and other projects [25, 26]. This method has high requirements on engineering geological conditions and mechanical reliability, and different operating conditions should also adapt to different shield ways. There are many researches on shield technology and construction safety in civil engineering field. This section makes a literature review to clarify the deficiencies of existing research.

### 2.1. Technology Research on Slurry Balancing Shield

Shield construction uses machine to excavate and lining tunnel. It can generally divide into pneumatic shield, slurry pressure shield, earth pressure balance shield, mixed shield, and so on. In the process of shielding, the working face relies on slurry pressure to balance the water pressure to obtain stability. Slurry pressure mainly plays a supporting role, and it is always greater than groundwater pressure, thus forming an outward hydraulic gradient, which is the basic condition for maintaining working face stability [27, 28]. Composition of modern slurry balancing shield machine is shown in Figure 1. The existing research on shield construction technology mainly includes laboratory experiment, numerical simulation, field monitoring, and other methods, mainly studying shield construction performance under different geological conditions and soil-water mechanics in shield process.

Laboratory experiments mainly focus on stability of excavation surface and mechanical properties of filter cake in process of shielding, especially in case of large diameter excavation and complex stratum conditions [29–31]. When in process of shield, mud cakes often appear on the cutter head due to high viscosity of soil. Ref. [32] suggests adding dispersants to slurry to reduce viscosity of clay to prevent slurry from producing mud cakes. This experiment tested basic properties of slurry, and the potential of dispersant to reduce mud cakes was investigated by mixing test and viscosity test. Ref. reference [33] uses a self-designed grout penetration device to carry out the cake forming experiment of different grout ratios in circular gravel stratum, to study the influence of grout-specific gravity, viscosity, and grouting pressure on infiltration water amount and cake forming time, so as to achieve the best state of filter cakes. Similarly, reference [34] studied the effect of seawater intrusion on slurry and filter cake properties during shield construction of undersea tunnel by laboratory experiment. Besides, reference [35] studied the formation mechanism and mechanical properties of filter cake for large diameter shield excavation through microscopic experiments.

Numerical simulation and field monitoring are mainly used to verify the stability of soil structure, the soil-water coupling effect, the applicability of shield method, and so on [36–40]. Reference [36] developed a visual management platform for shield construction based on Web-GIS server. The system has realized functions of data management, 2D and 3D visualization, geospatial analysis, and real-time monitoring. Ref. [41] developed a lining structure detection system, which uses multiple CCD cameras to obtain high-resolution image information of tunnel surface, and uses intelligent analysis method to identify and quantify lining damage. Ref. [42] used numerical simulation to simulate formation process of working face fracture caused by slurry pressure, and they considered the coupling of stress distribution, fluid flow, and fracturing process. Besides, some scholars have studied the operation process of shield tunneling from a microscopic perspective by using meso-mechanics [43], and the deformation of foundation under different stress paths [44].

### 2.2. Risk Management of Shield Construction

At present, researches on safety risk management of tunnel shield construction are mainly qualitative analysis, most of which focus on a specific link in the construction process. Main research methods are mathematical modeling and numerical analysis. Reference [45] compared advantages and disadvantages of AHP, BN, and FTA risk assessment models and constructed a risk evaluation network by analyzing causal relationships between risk factors and events. Meanwhile, he proposed a causal network matrix model suitable for tunnel construction safety risk analysis. In order to predict settlement risk during shield excavation reference [46], we proposed a fuzzy hybrid method for coupling Bayesian network and bow-tie model. By integrating weighted expert opinions, probabilities of environmental faults, operation errors, and other faults are obtained, and settlement risk values evaluated systematically from multiple aspects. Stability of shield working face is very important for safety and risk management of shield tunneling, reference [47] and we proposed a predictive control system of shield chamber pressure based on particle swarm optimization and neural network model to prevent surface collapse. Face to preliminary design stage, Reference [48], used accident tree analysis to quantify TBM risks, and selected appropriate risk mitigation measures to ensure construction safety. Based on fuzzy entropy theory, reference [19] we established a comprehensive evaluation index system. In order to quantitatively analyze coupling degree of each index, according to the coupling degree theory, calculation model of coupling degree is established to monitor safety risks of shield tunnel construction. In addition, rough set theory, cloud model, and index system analysis methods are often used in tunnel shield risk analysis [18, 49].

Overall, current research on slurry balancing shield construction is still technology-oriented, mainly focus on specific problems such as geotechnical properties, working face stability, and filter cake effectiveness, and methods adopted are still mainly laboratory experiments and computer numerical simulation. Objects of risk analysis are mainly concrete type such as settlement risk and collapse risk, which is mainly calculated by mathematical method. This paper counts slurry balancing shield process as an integrative system, and construction risk factors are divided into “human-machine-material-method-environment” five major categories, then using modified AHP combined with FSE to form an assessment model and calculate certain risk value. The result is a supplement to current risk management research.

## 3. Risk Assessment Model for Shield Construction

### 3.1. Establishment of Risk Evaluation Index System

Risk assessment index usually comes from analysis of construction process. The whole process of slurry balancing shield tunneling can be generally divided into five stages, that is, preconstruction preparation, working well and shield preparation, shield construction, internal and auxiliary structure construction, and cleaning and recovery. Main contents of each stage are shown in Table 1.

The third-stage shield construction can be divided into site layout, preconstruction preparation, tunnel excavation, and synchronous construction according to the process, as shown in Figure 2.

Establishment of risk assessment index system is the key step for risk evaluation. According to the way of stratification and grading of index system, the system is divided into target layer and index layer. Target layer is risk of slurry shield construction. According to the characteristics of tunnel construction, risk factors are divided into five types: human, machine, material, method, and environment. Risk evaluation is an integrated analysis of these five risk types. Flowchart of indicator system establishment is shown in Figure 3.

According to above process, a questionnaire survey was conducted for the selection of risk indicators. We made an index screening questionnaire and asked 20 participating experts whether each index needs to be selected, the reasons for not selecting, and the indicators that need to be added in detail. These 20 experts all come from tunnel construction industry and have redundant experiences on construction risk management. Based on expert investigations, risk evaluation indicator system of slurry balancing shield construction was formed as shown in Table 2.

In this evaluation system, there are 5 indicators at first level, 12 indicators at second level, and 29 indicators at third level, and third-level index is the basic index.

### 3.2. AHP-FSE Risk Assessment Model

#### 3.2.1. Analytic Hierarchy Process

Analytic hierarchy process (AHP) is a system engineering modeling method. Its essence is to solve multilevel, multi-objective, semistructured, and unstructured problems by determining the weight of indicators at all levels, which is widely used in engineering risk analysis. It usually includes these following steps:

*(1)* Establish hierarchical model: the first step of AHP is to establish hierarchical model, which is to decompose the overall objective layer by layer and form an evaluation system composed of a variety of elements. It is generally composed of target layer, criterion layer, and index layer.

(*2)* Construct judgment matrix: the hierarchical model reflects dominance relationship between adjacent elements at different levels. According to this relationship, all elements are compared in pairs and scored according to the 1–9 scale method, as shown in Table 3, to form a judgment matrix.

The form of the judgment matrix is as follows:

(1) $$\begin{array}{c} B=\left[\begin{array}{cccc} b_{11} & b_{12} & \cdots & b_{1n}\\ b_{21} & b_{22} & \cdots & b_{2n}\\ \vdots & \vdots & \vdots & \vdots \\ b_{n1} & b_{n2} & \cdots & b_{nn} \end{array}\right]. \end{array}$$

*b*_*ij*_=*w*_*i*_/*w*_*j*_, is the ratio of influence of *w*_*i*_ to *w*_*j*_ on factor *x.* The judgment matrix is a special matrix whose elements satisfy the following conditions:

(2) $$\begin{array}{c} b_{ii}=1,\\ b_{ii}=\frac{1}{b_{ji}},\\ b_{ji}=\frac{b_{ik}}{b_{jk}}. \end{array}$$

Since the judgment matrix is obtained by experts' scoring of the evaluation object, it is subjective and difficult to guarantee its accuracy. Therefore, it is necessary to check the consistency of the matrix to determine whether it meets the accuracy requirements. The inspection steps are as follows:

(1) Calculate maximum eigenvalue *λ*_max_ of judgment matrix.
(2) Calculate consistency index C.I. and the consistency ratio C.R:
  (3) $$\begin{array}{c} C.I=\frac{\lambda_{\max}-n}{n-1}, \end{array}$$
  (4) $$\begin{array}{c} C.R=\frac{C.I.}{R.I.}, \end{array}$$
where *R.I*. is average random consistency indicator, which can be found in Table 4. When *C.R*. value below 0.1, matrix B has good consistency.
(3) Calculate Index Single SortSorting refers to calculating the weight of lower element to an upper element when the judgment matrix B has good consistency. In fact, the sort calculation is to find the maximum nonzero eigenvalue of judgment matrix and its corresponding eigenvector, generally using the root method:
  (1) Take product of each row of judgment matrix *M*_*i*_:
    (5) $$\begin{array}{c} M_{i}=\prod_{j=1}^{n}b_{ij}\;i=1,2,3,\cdots n. \end{array}$$
  (2) Calculate the n^th^ root of *Mi*:
    (6) $$\begin{array}{c} W={\left(\prod_{j=1}^{n}b_{ij}\right)}^{\frac{1}{n}},\;i=1,2,3,\cdots n. \end{array}$$
  (3) The normalization of *W* is the weight.
  (4) Calculate maximum eigenvalue *λ*_max_:
    (7) $$\begin{array}{c} \lambda_{\max}=\frac{1}{n}\sum_{i=1}^{n}\frac{{\left(Bw\right)}_{i}}{w_{i}}. \end{array}$$
(4) Calculate the Total Ranking and Consistency. Total ranking refers to the relative weight of each element to total target. The total sort should be calculated from top to bottom. It is assumed that single-ranking weight vector A^(*k*)^ in *k* layer for (k-1) layer and the total ranking vector W^(k−1^) of the (k-1) layer relative to the total target are known:
  (8) $$\begin{array}{c} A^{\left(k\right)}=\left[\begin{array}{cccc} w_{11}^{\left(k\right)} & w_{12}^{\left(k\right)} & \cdots & w_{1m}^{\left(k\right)}\\ w_{21}^{\left(k\right)} & w_{22}^{\left(k\right)} & \cdots & w_{2m}^{\left(k\right)}\\ \vdots & \vdots & \vdots & \vdots \\ w_{n1}^{\left(k\right)} & w_{n1}^{\left(k\right)} & \cdots & w_{nm}^{\left(k\right)} \end{array}\right]. \end{array}$$
Then, the total sort of the layer K is *W*^(*k*)^=*A*^(*k*)^ · *W*^(*k* − 1)^.
Total ranking consistency test of layer K is calculated as follows:
  (9) $$\begin{array}{c} C.R.^{\left(k\right)}=\frac{C.I.^{\left(k\right)}}{R.I.^{\left(k\right)}},\\ C.I.^{\left(k\right)}=\left(C.I._{1}^{\left(k\right)},C.I._{2}^{\left(k\right)},\cdots ,C.I._{n}^{\left(k\right)}\right)W^{\left(k-1\right)},\\ R.I.^{\left(k\right)}=\left(R.I._{1}^{\left(k\right)},R.I._{2}^{\left(k\right)},\cdots ,R.I._{n}^{\left(k\right)}\right)W^{\left(k-1\right)}. \end{array}$$
  when C.R. < 0.1, the total sorting has good consistency.

#### 3.2.2. Fuzzy Synthetic Evaluation

Fuzzy synthetic evaluation method weakens the influence of expert subjective judgment and can effectively analyze fuzzy concepts that are difficult to be quantified such as tunnel shield construction risk. FSE mainly divided into these following steps:

*(1)* Determine factor set *U*: factor set *U*=(*u*_1_, *u*_2_, ⋯, *u*_*m*_.), 1,2, ⋯*m* is a set that reflects factors that have impact on evaluation object and is generally determined by risk evaluation index system.

*(2)* Establish evaluation set *V*: evaluation set *V*=(*v*_1_, *v*_2_, ⋯, *v*_*m*_), 1,2, ⋯*m* is a set reflecting the judgment results made by experts on evaluation object.

*(3)* Determine factor weight vector *W*: factor weight vector *W*=(*w*_1_, *w*_2_, ⋯, *w*_*m*_), 1,2, ⋯*m* reflects the importance of each factor, that is, the weight of layer K factor to layer K-1 factor, which is calculated by analytic hierarchy process.

*(4)* Calculate evaluation matrix *R*: the evaluation matrix *R* is to evaluate the last layer of factors in index system by inviting experts to use comments in the evaluation set V, and determine the membership degree of each factor. General form of evaluation matrix is as follows:

(10) $$\begin{array}{c} R=\left[\begin{array}{cccc} r_{11} & r_{12} & \cdots & r_{1n}\\ r_{21} & r_{22} & \cdots & r_{2n}\\ \vdots & \vdots & \vdots & \vdots \\ r_{m1} & r_{m2} & \cdots & r_{mn} \end{array}\right], \end{array}$$

where *r*_*ij*_ represents the membership degree of factor *U*_*i*_ to comment *V*_*i*_.

*(5)* Calculate evaluation results: according to factor weight vector W and evaluation matrix *R*, then calculate risk value of last level factors in index system, the evaluation formula is as follows:

(11) $$\begin{array}{c} A=W\circ R. \end{array}$$

where ″°″ is an operator, commonly include principal factor or average weighted determination. Since the final evaluation result is an vector, risk level of project can be determined according to principle of maximum membership degree. In this paper, slurry balancing shield construction risk assessment is mainly calculated based on fuzzy synthetic evaluation method, and the evaluation steps are shown in Figure 4.

## 4. Case Study

### 4.1. Project Overview

River-crossing tunnel project of Nanjing Metro Line 3 is from Liuzhou East Road station to Shangyuanmen station. This project adopts slurry balancing shield construction. The tunnel crosses the Yangtze river, and engineering geology and hydrogeology conditions are complex, so construction process is difficult and under uncertain risks. Total length of the tunnel is about 3300 m.  Figure 5 shows the geographical location of this project.

The tunnel adopts a Ф11570-mm slurry shield machine for construction, tunnel lining structure's outer diameter is 11200 mm, inner diameter is 10200 mm, lining thickness is 500 mm, and ring width is 2000 mm. The tunnel lining adopts general wedge segment and staggered assembling method. Lining rings are divided into 8 pieces, namely, 5 standard blocks, 2 connecting blocks, and 1 top sealing block. The workload of shield tunneling is shown in Table 5.

The tunnel passes through a number of residential buildings and other construction structures. Soil conditions are mainly silt sand, accounting for more than 50% of the excavated soil. The groundwater along the line is mainly pore water of loose rock and bedrock water. The variation of the water table is mainly affected by atmospheric precipitation, and the annual variation range is generally between 0.5 and 1.0 m.

### 4.2. Safety Risk Assessment of Slurry Shield Construction

#### 4.2.1. Determination of Indicator Weights

Considering subjective factors, 10 tunnel experts were invited to score the risk index system, and then, analytic hierarchy process was used to calculate weight of each questionnaire. These 10 experts are all from this project, and they are all senior managers with more than 10 years working experiences. Finally, average weight of all the questionnaires was taken as the calculation result. Take scoring result of an expert as a case to illustrate.

*(1) First-layer index weight*.  Table 6 lists scores of first-layer indicators. The judgment matrix of the first-layer index is as follows:

(12) $$\begin{array}{c} B=\left[\begin{array}{ccccc} 1 & 2 & 3 & 2 & \frac{1}{3}\\ \frac{1}{2} & 1 & 2 & \frac{1}{2} & \frac{1}{5}\\ \frac{1}{3} & \frac{1}{2} & 1 & \frac{1}{3} & \frac{1}{6}\\ \frac{1}{2} & 2 & 2 & 1 & \frac{1}{4}\\ 3 & 5 & 6 & 4 & 1 \end{array}\right] \end{array}$$

Weight vector $W=\left(\begin{array}{ccccc} 0.202 & 0.096 & 0.060 & 0.144 & 0.498 \end{array}\right)$, obtained from equations (5) and (6). The maximum eigenvalue *λ*_max_ = 5.099, R.I. = 1.12, C.I. = 0.0248, *C*.*R*.=(*C*.*I*./*R*.*I*.)=(0.0248/1.12)=0.0221=0.1; therefore, the judgment matrix has good consistency.

*(2) Second-layer index weight*

(a) Weight vector of personnel risk
Judgment matrix of personnel risk:
  (13) $$\begin{array}{c} B_{1}=\left[\begin{array}{ccc} 1 & 3 & 5\\ \frac{1}{3} & 1 & 2\\ \frac{1}{5} & \frac{1}{2} & 1 \end{array}\right],\\ W_{1}=\left(\begin{array}{ccc} 0.648 & 0.230 & 0.122 \end{array}\right)\lambda_{\text{max}}=3\text{.}003\text{, R.I.}=\text{0.}58\text{, C.I.}=\text{0.}0015\text{, C.R.}=\frac{\text{C.I.}}{\text{R.I.}}=\frac{\text{0.}0015}{\text{0.}58}=\text{0.}0026<\text{0.}1\text{.} \end{array}$$
Using the same method, it can be obtained as follows:
(b) Weight vector of mechanical risk: $W_{2}=\left(\begin{array}{cc} 0.33 & 0.67 \end{array}\right)$,
(c) Weight vector of material risk: $W_{3}=\left(\begin{array}{cc} 0.67 & 0.33 \end{array}\right)$,
(d) Weight vector of method risk: $W_{4}=\left(\begin{array}{cc} 0.67 & 0.33 \end{array}\right)$,
(e) Weight vector of environmental risk: $W_{4}=\left(\begin{array}{ccc} 0.594 & 0.249 & 0.157 \end{array}\right)$.

*(3) Third-layer index weight*

(a) Weight of professional skills and experience
  (14) $$\begin{array}{c} B_{11}=\left[\begin{array}{cccccc} 1 & \frac{1}{3} & 1 & 2 & \frac{1}{3} & \frac{1}{3}\\ 3 & 1 & 3 & 4 & \frac{1}{2} & 2\\ 1 & \frac{1}{3} & 1 & 2 & \frac{1}{3} & \frac{1}{2}\\ \frac{1}{2} & \frac{1}{4} & \frac{1}{2} & 1 & \frac{1}{4} & \frac{1}{3}\\ 3 & 2 & 3 & 4 & 1 & 1\\ 3 & \frac{1}{2} & 2 & 3 & 1 & 1 \end{array}\right], \end{array}$$

$W_{11}=\left(\begin{array}{cccccc} 0.108 & 0.253 & 0.096 & 0.059 & 0.284 & 0.201 \end{array}\right),\;\lambda_{\text{max}}=6\text{.}502\text{, R.I.}=1\text{.}12\text{, C.I.}=\text{0.}1004\text{, C.R.}=\left(\text{C.I.}/\text{R.I.}\right)=\left(\text{0.}1004/1\text{.}12\right)\text{0.}09<\text{0.}1$ . The judgment matrix has good consistency. Using same method, the weight vectors of other indexes in third layer can be obtained. All questionnaires were processed in accordance with the above process, and the average value of each index weight was obtained, as shown in Table 7.

In first layer, weights of personnel risk, mechanical risk, and environmental risk are larger than others. Therefore, when planning risk prevention, project managers should first take personnel, machinery, and environmental risks into consideration.

#### 4.2.2. Fuzzy Synthetic Evaluation

*(1) Determine factor set U and evaluation set V*. *U*=(*u*_1_, *u*_2_, ⋯, *u*_*m*_), 1,2, ⋯*m* corresponds to third-level index in evaluation index system, *V*=(*v*_1_, *v*_2_, ⋯, *v*_*m*_), 1,2, ⋯*m* =(large, relatively large, normal, relatively small, small).

*(2) Single-factor evaluation results*. 20 experts were invited to fill in the \questionnaire to conduct a single-factor evaluation on risk of third-level indicators in the index system, and frequency of each indicator being selected was counted. The evaluation matrix was established according to the results shown in Table 8.

*(3) First-level evaluation*. The weight of the first-layer index and the single factor evaluation value can get the result of the first-level fuzzy synthetic evaluation.

(15) $$\begin{array}{c} A_{1}=W_{11}\circ R_{11}=\left(\begin{array}{cccc} 0.38 & 0.20 & 0.18 & 0.24 \end{array}\right)\left[\begin{array}{ccccc} 0 & 0.4 & 0.15 & 0.2 & 0.25\\ 0 & 0 & 0 & 0.3 & 0.7\\ 0 & 0.1 & 0.25 & 0.15 & 0.5\\ 0.3 & 0.3 & 0.1 & 0.15 & 0.15 \end{array}\right]=\left(\begin{array}{ccccc} 0.065 & 0.2145 & 0.1875 & 0.2265 & 0.3065 \end{array}\right). \end{array}$$

where *W*_*11*_ is the weight vector of *A*_*1*_, and *R*_*11*_ is the judgment matrix of *A*_*1*_. In the same way, A2 to E3 should be add in single display math and that no should be add in matrix format

(16) $$\begin{array}{c} A_{2}=\begin{array}{ccccc} \left(0\right. & 0 & 0.274 & 0.279 & \left.0.447\right) \end{array},\\ A_{3}=\begin{array}{ccccc} \left(0.108\right. & 0.072 & 0.15 & 0.26 & \left.0.41\right) \end{array},\\ B_{1}=\begin{array}{ccccc} \left(0\right. & 0.011 & 0.154 & 0.393 & \left.0.445\right), \end{array}\\ B_{2}=\begin{array}{ccccc} \left(0.0155\right. & 0.0155 & 0.031 & 0.23 & \left.0.708\right), \end{array}\\ C_{1}=\begin{array}{ccccc} \left(0.0005\right. & 0.011 & 0.0615 & 0.269 & \left.0.653\right) \end{array},\\ C_{2}=\begin{array}{ccccc} \left(0.049\right. & 0.095 & 0.335 & 0.1805 & \left.0.305\right) \end{array},\\ D_{1}=\begin{array}{ccccc} \left(0.013\right. & 0.059 & 0.168 & 0.256 & \left.0.495\right) \end{array},\\ D_{2}=\begin{array}{ccccc} \left(0\right. & 0 & 0.042 & 0.291 & \left.0.633\right) \end{array},\\ E_{1}=\begin{array}{ccccc} \left(0.009\right. & 0.0456 & 0.1155 & 0.198 & \left.0.636\right) \end{array},\\ E_{2}=\begin{array}{ccccc} \left(0\right. & 0.021 & 0.0455 & 0.206 & \left.0.7265\right) \end{array},\\ E_{3}=\begin{array}{ccccc} \left(0.19\right. & 0.021 & 0.094 & 0.198 & \left.0.332\right) \end{array}. \end{array}$$

*(4) Second-level evaluation*

(17) $$\begin{array}{c} A=W_{1}\circ R_{1}\left(\begin{array}{ccc} 0.56 & 0.24 & 0.20 \end{array}\right)\left[\begin{array}{ccccc} 0.065 & 0.2145 & 0.1875 & 0.2265 & 0.3065\\ 0 & 0 & 0.274 & 0.279 & 0.447\\ 0.108 & 0.072 & 0.15 & 0.26 & 0.41 \end{array}\right]=\left(\begin{array}{ccccc} 0.058 & 0.13452 & \;0.20076 & 0.17785 & 0.36092 \end{array}\right) \end{array}$$

where *W*_*1*_ is the weight vector of index A, and *R*_*1*_ is the judgment matrix composed of the first-level fuzzy comprehensive evaluation results of index *A*_*1*_ and *A*_*2*_. In the same way,

$B=W_{2}\circ R_{2}=\left(\begin{array}{ccccc} 0.00915 & 0.0137 & 0.08143 & 0.29683 & 0.60017 \end{array}\right)$ ,

$C=W_{3}\circ R_{3}=\left(\begin{array}{ccccc} 0.02378 & 0.05132 & 0.19278 & 0.22652 & 0.503 \end{array}\right)$ ,

$D=W_{4}\circ R_{4}=\left(\begin{array}{ccccc} 0.00442\; & 0.02006\; & 0.08484 & 0.27976 & 0.60786 \end{array}\right)$ ,

$E=W_{5}\circ R_{5}=\left(\begin{array}{ccccc} 0.06313 & 0.030635 & 0.093655 & 0.19976 & 0.56167 \end{array}\right)$ .

*(5) Third-level evaluation*

(18) $$\begin{array}{c} Z=W\circ R=\left(\begin{array}{ccccc} 0.27 & 0.25 & 0.14 & 0.11 & 0.23 \end{array}\right)\left[\begin{array}{ccccc} 0.058 & 0.13452 & 0.20076 & 0.17785 & 0.36092\\ 0.00915 & 0.0137 & 0.08143 & \;0.29683 & 0.60017\\ 0.02378 & 0.05132 & 0.19278 & 0.22652 & 0.503\\ 0.00442 & 0.02006 & 0.08484 & 0.27976 & 0.60786\\ 0.06313 & 0.030635 & \;0.093655 & 0.19976 & 0.56167 \end{array}\right]=\left(\begin{array}{ccccc} 0.04096 & 0.06357 & 0.13711 & 0.21912 & 0.50052 \end{array}\right). \end{array}$$

Z is the risk evaluation vector of the cross-river tunnel. According to the principle of maximum membership degree, 0.50052 is taken as the highest value in the evaluation vector, corresponding to “small” in the evaluation set; that is, the risk of this project is small and the safety situation is good.

#### 4.2.3. Evaluation Results Analysis

As shown in above evaluation results, the overall risk level of case project is small and in a safe state, but risk level of some indicators is relatively high, so corrective measures need to be formulated to strengthen prevention. The personnel risk is very small, indicating that overall staff quality of this project is good. From material perspective, risk of other basic indicators is small except dimensional discrepancy and stacking condition, and this requires strict inspection of material acceptance. The overall risk of construction environment, mechanical, and method is in safe state. All basic indicators are at relatively light risk level, indicating that safety management of this project is successful.

## 5. Risk Mitigation Measures

Safety risk identification of slurry balancing shield mainly focuses on five aspects of whole construction process: human-machine-material-method-environment. AHP-FSE analysis shows that human operation, mechanical equipment selection, and construction environment could have a relatively high probability to cause safety accidents, so risk mitigation and response measures should focus on these aspects. From management and economic perspectives, risk mitigation measures corresponding to slurry shield construction are proposed. Since shield construction is with strong dependence on mechanical equipment, the reliability and applicability of shield machine can directly determine the quality of construction. Therefore, this paper makes a detailed analysis of shield machine selection, aim to alleviating construction safety risks by improving machine adaptability.

### 5.1. Management and Economic Measures

Due to complex mechanical equipment and construction process, it is necessary to organize and manage project according to different situations. Therefore, it is of great significance to clarify project planning and management objectives and carry out systematic management, then scientifically organize workers' education and training, site management, and hidden accidents' investigation. Through adoption of “planning, implementation, inspection, and improvement” cycle safety management mode, use of safety production standardization system, and institutionalized management, it can better promote continuous improvement of safety production and formation of safety culture. Economic measures are another important way to realize risk mitigation. Risk management can be carried out through whole life-cycle project management, establishment of reward and punishment mechanism, occupational health, and safety investment. Management and economic measures are shown in Figure 6.

### 5.2. Technical Measures: Shield Machine Selection

Selection of slurry shield machine is mainly based on design documents, in accordance with principles of applicability, reliability, advancement, and economy. Shield machine selection generally needs to meet the following requirements:

  Basis 1: Engineering geology (mainly analyzing the distribution of soil layer, soil property, and particle size in shield tunnel interval),
  Basis 2: Engineering environment (mainly analyzing shield tunnel crossing structures),
  Basis 3: Requirements for long-distance crossing rivers and seas,
  Basis 4: Condition of large buried depth and high water pressure,
  Basis 5: Synchronous construction requirements.

Shield machine selected for different projects should be designed according to characteristics of the project, especially considering hydrogeological conditions, surrounding environmental conditions, long-distance underwater excavation, and other major risk points. Critical consideration should be given to the cutter head structure, driving system, synchronous grouting, shield tail sealing system, and other aspects. It is particularly effective to avoid construction safety risks by selecting correct equipment for shield construction. The matching relationship between shield machine performance and engineering characteristics is shown in Table 9.

## 6. Discussion and Conclusion

### 6.1. Discussion

Slurry balancing shield construction has been widely used in cross-river tunnel construction because of its strong ability to control working face stability. However, the technology is not mature enough and the shield equipment research is still in optimization stage. In terms of risk management, compared with other municipal projects, construction quantity of slurry shield tunnel still occupies a small share. Therefore, there are still many construction safety risks that have not been discovered and need to be continuously supplemented in the process of subsequent research. The risk evaluation system proposed in this paper still has room for modification.

Risk management is a complex system engineering, which should be considered from the perspective of the whole project life cycle and all stakeholders. However, due to the complexity of construction technology and the complicated process, it is difficult to systematically integrate the whole construction process. At present, research on the whole life cycle and critical risk control measures and experiences are still insufficient, and few companies can carry out slurry shield construction. The construction process still mainly relies on experienced engineers to control, identify, and manage risks, and it is necessary to make their tacit knowledge of critical risk management explicit.

Due to particularity and complexity of construction, conventional qualitative and quantitative analyses are limited for safety risk analysis, which cannot be comprehensively analyzed. Therefore, the establishment of risk analysis index system is particularly important. Existing technical research is aim to solve problems of specific operation works, but for the overall safety control, it is necessary to integrate the construction process and build a risk analysis index system that can represent the whole construction life cycle.

## 7. Conclusion

Taking construction safety risk as research goal, this paper objectively analyzes cases of different types of large-diameter slurry balancing shield tunnel, summarizes the slurry shield construction process, and then divides construction risk into five categories of “human-machine-material-method-environment” from the perspective of whole project life cycle. This paper innovatively proposed the model of analytic hierarchy process combined with fuzzy synthetic evaluation to identify and evaluate safety risks of slurry balancing shield construction. Finally, we use a case study to verify the risk analysis model and put forward risk prevention measures for slurry balancing shield construction [38]. Main conclusions of this paper are as follows:

1. Using analytic hierarchy process and fuzzy synthetic evaluation method, this paper constructs a safety risk evaluation model of slurry balancing shield and modified the traditional calculation method. Weight of indicators is calculated by analytic hierarchy process, and the evaluation matrix is constructed by fuzzy evaluation method. This paper combines evaluation set and maximum membership degree to output risk calculation results. Combination of subjective and objective methods improves the accuracy of calculation results.
2. Through index weight calculation, it can be seen that personnel risk, mechanical equipment risk, and environmental risk accounts for a large proportion in the overall evaluation system. Among personnel risks, professional skills and experience have the largest weight. When selecting workers, management staff should first pay attention to their working experiences. Among mechanical risks, the qualified rate of maintenance has a relatively high risk, so it is necessary to maintain the machinery regularly and strictly check the quality before entering the site. In the material risk, the physical property risk value is larger than others, so quality control should be paid more attention. In the method risk, drawings change may result in accidents; therefore, engineering drawings need to be carefully reviewed. In the environmental risk, geological conditions are more risky. For areas with poor geological conditions, measures should be taken to reinforce soil layer.
3. This paper takes Nanjing Metro Line 3 cross-river tunnel project as a case study, verified the effectiveness of proposed risk evaluation method based on AHP and FSE, and systematically expounded how to identify, evaluate, and precontrol risks in slurry balancing shield construction. Related risk mitigation measures are put forward from aspects of management, economic, and technology, and parameter selection of shield machine is discussed in detail. The research results provide a reference for slurry shield construction under different working conditions in the future.

## Figures and Tables

**Figure 1:** Composition of slurry shield machine.

**Figure 2:** Flowchart of slurry balancing shield tunneling.

**Figure 3:** Indicator system establishment flowchart.

**Figure 4:** Flowchart of slurry shield tunnel construction risk assessment.

**Figure 5:** Layout of Nanjing Metro Line 3 crossing river tunnel project.

**Figure 6:** Management and economic measures for risk mitigation.

**Table 1:** Construction stage division and content of slurry balancing shield.

Stage division	Overview	Main construction operation content
Stage I	Preconstruction preparation	(1) Site preparation. Construction site, living and production facilities, and pipeline relocation (2) Technical preparation. Construction organization and scheme, and pile measurement (3) Human, machine, and material preparation. Construction team, facility inspection, and materials inspection

Stage II	Working well and shield preparation	(1) Enclosure, drainage, and support for working well (2) Shield-related preparation shield machine transportation, pipe transportation, and slurry separation field

Stage III	Shield construction	Shield machine installation, test tunneling, and normal operation

Stage IV	Internal and auxiliary structure	(1) Inner structure (2) Mechanical and electrical (3) Accessory structure

Stage V	Clean and recovery	Internal structure cleaning, site cleaning, traffic, and greening restoration

**Table 2:** Risk evaluation index system for slurry balancing shield.

Target layer	First layer	Second layer	Third layer
Risk of slurry shield construction	Personnel risk (A)	Professional skills and experience (A1)	Working experience (A11)
			Safety skills (A12)
			Emergency capacity (A13)
			Safety consciousness (A14)
		Physical condition (A2)	Working strength (A21)
			Physical health (A22)
		Mental health status (A3)	Sense of discipline (A31)
			Working pressure (A32)
	Mechanical risk (B)	Mechanical use status (B1)	Mechanical failure condition (B11)
			Mechanical aging condition (B12)
			Mechanical wear condition (B13)
		Mechanical qualification status (B2)	Qualification rate of installation (B21)
			Qualification rate of maintenance (B22)
	Material risk (C)	Material quality status (C1)	Physical property (C11)
			Dimensional discrepancy (C12)
		Material storage status (C2)	Storage conditions (C21)
			Stacking condition (C22)
	Method risk (D)	Security system (D1)	Integrity degree (D11)
			Executive capacity (D12)
			Implementation effect (D13)
		Construction schemes (D2)	Working method (D21)
			Drawings change (D22)
	Environmental risk (E)	Geological environment (E1)	Geological conditions (E11)
			Geological disaster situation (E12)
		Social environment (E2)	Surrounding traffic conditions (E21)
			Settlement level of surrounding buildings (E22)
			Underground pipeline relocation (E23)
		Site environment (E3)	Safety facilities (E31)
			Water pollution (E32)

**Table 3:** Scaling score table.

Scale	Definition
1	*W*_*i*_ is as important as *W*_*j*_
3	*W*_*i*_ is slightly important than *W*_*j*_
5	*W*_*i*_ is more important than *W*_*j*_
7	*W*_*i*_ is strongly important than *W*_*j*_
9	*W*_*i*_ is extremely important than *W*_*j*_
2, 4, 6, 8	Intermediate value
Reciprocal	*b*_*ji*_=*b*_*j*_/*b*_*i*_, *b*_*ji*_=1/*b*_*ij*_

**Table 4:** Average random consistency index values.

*n*	2	3	4	5	6	7	8	9
*R*.*I*.	0	0.58	0.9	1.12	1.24	1.32	1.44	1.45

**Table 5:** Shield tunneling workload.

Number	Contents	Unit workload (step)	Total workload	Remarks
1	Shield distance	2 m	3353.945 m	Whole tunnel
2	Excavated Earth volume	211.37 m^3^	352622.8 m^3^	Whole tunnel
3	Synchronous grouting	22.92 m^3^∼25.79 m^3^	38438.6 m^3^∼43243.4 m^3^	160% to 180% of theoretical building gap (theoretical 14.33 m^3^/step)
4	Replication slurry	—	—	Depending on the actual situation

**Table 6:** First-layer index scores.

*w*_*j*_	*W*_*i*_				
	Personnel risk	Mechanical risk	Material risk	Method risk	Environmental risk
Personnel risk	1	2	3	2	1/3
Mechanical risk	1/2	1	2	1/2	1/5
Material risk	1/3	1/2	1	1/3	1/6
Method risk	1/2	2	3	1	1/4
Environmental risk	3	5	6	4	1

**Table 7:** Weight of safety risk assessment index system of slurry balancing tunnel.

Target layer	First layer	Weight	second layer	Weight	The third layer	Weight
Risk of slurry shield construction	Personnel risk (A)	0.27	Professional skills and experience (A1)	0.56	Working experience (A11)	0.38
					Safety skills (A12)	0.20
					Emergency capacity (A13)	0.18
					Safety consciousness (A14)	0.24
			Physical condition (A2)	0.24	Working strength (A21)	0.59
					Physical health (A22)	0.41
			Mental health status (A3)	0.20	Sense of discipline (A31)	0.66
					Working pressure (A32)	0.34
	Mechanical risk (B)	0.25	Mechanical use status (B1)	0.41	Mechanical failure condition (B11)	0.48
					Mechanical aging condition (B12)	0.22
					Mechanical wear condition (B13)	0.30
			Mechanical qualification status (B2)	0.59	Qualification rate of installation (B21)	0.42
					Qualification rate of maintenance (B22)	0.58
	Material risk (C)	0.14	Material quality status (C1)	0.52	Physical property (C11)	0.63
					Dimensional discrepancy (C12)	0.37
			Material storage status (C2)	0.48	Storage conditions (C21)	0.46
					Stacking condition (C22)	0.54
	Method risk (D)	0.11	Security system (D1)	0.34	Integrity degree (D11)	0.26
					Executive capacity (D12)	0.44
					Implementation effect (D13)	0.30
			Construction schemes (D2)	0.66	Work method (D21)	0.42
					Drawings change (D22)	0.58
	Environmental risk (E)	0.23	Geological environment (E1)	0.47	Geological conditions (E11)	0.65
					Geological disaster situation (E12)	0.35
			Social environment (E2)	0.22	Surrounding traffic conditions (E21)	0.09
					Settlement level of surrounding buildings (E22)	0.49
					Underground pipeline relocation (E23)	0.42
			Site environment (E3)	0.31	Safety facilities (E31)	0.63
					Water pollution (E32)	0.37

**Table 8:** Single-factor evaluation results.

Factors	Risk level				
	Large	Relatively large	Normal	Relatively small	Small
Working experience	0	0.4	0.15	0.2	0.25
Safety skills	0	0	0	0.3	0.7
Emergency capacity	0	0.1	0.25	0.15	0.5
Safety consciousness	0.3	0.3	0.1	0.15	0.15
Working strength	0	0	0.4	0.3	0.3
Physical health	0	0	0.1	0.25	0.65
Sense of discipline	0	0	0.15	0.35	0.5
Working pressure	0.3	0.2	0.15	0.1	0.25
Mechanical failure condition	0	0	0.15	0.3	0.55
Mechanical aging condition	0	0.05	0.1	0.45	0.4
Mechanical wear condition	0	0	0.2	0.5	0.3
Qualification rate of installation	0	0	0	0.35	0.65
Qualification rate of maintenance	0	0	0	0.25	0.75
Physical property	0	0	0	0.35	0.65
Dimensional discrepancy	0.05	0.1	0.4	0.25	0.2
Storage conditions	0	0.05	0.2	0.25	0.5
Stacking condition	0.1	0.15	0.5	0.1	0.15
Integrity degree	0	0	0.25	0.3	0.45
Executive capacity	0.05	0.1	0.2	0.2	0.45
Implementation effect	0	0.05	0.05	0.3	0.6
Working method	0	0	0.1	0.35	0.55
Drawings change	0	0	0	0.25	0.75
Geological conditions	0.25	0.3	0.1	0.2	0.15
Geological disaster situation	0	0	0	0.05	0.95
Surrounding traffic conditions	0	0	0.05	0.15	0.8
Settlement level of surrounding buildings	0	0	0	0.05	0.95
Underground pipeline relocation	0	0.05	0.1	0.4	0.45
Safety facilities	0.25	0.25	0.15	0.2	0.15
Water pollution	0	0.05	0.15	0.45	0.35

**Table 9:** Shield machine performance requirements.

Basic rules	Performance requirements of shield machine
(1) Engineering geology	(1) The size of shield machine must conform to the tunnel size. (2) The cutters of shield tunneling must adapt to the harsh geological conditions

(2) Engineering environment	(3) Shield machine has air pressure (or normal pressure) knife change conditions, and fully equipped. (4) Equipped with machine to reinforce the working surface soil.

(3) Long distance across rivers and seas	(5) The cutter head is equipped with a mixer, and pipe entrance is equipped with a crusher. (6) The antideformation ability of shield tail should meet the construction requirements (7) Shield assembly performance is efficient and matches with the general segment

(4) Large buried depth and high water pressure	(8) The normal service life of cutter head bearing and sand seal system should meet the requirements. (9) The sealing capacity of the soil and sand sealing system should meet the requirements. (10) The sealing capacity of shield tail seal shall meet the requirements

(5) Synchronous construction requirements	(11) Single liquid mortar is used for synchronous grouting, and the shield machine should have corresponding devices for grouting. (12) Frame system needs to meet the requirements of shield equipment layout.

## Data Availability

The data used to support the findings of this study are available from the corresponding author upon reasonable request.
